# Metaphoric Function and Emotional Cognition of English Loanwords in the Internet Environment

**DOI:** 10.1155/2022/1502959

**Published:** 2022-09-02

**Authors:** Hui Liu

**Affiliations:** Department of Foreign Language, Zhanjiang University of Science and Technology, Zhanjiang 524000, China

## Abstract

With the rapid development of society, the emergence and innovation of network buzzwords continue to emerge. On the rapidly changing social network platform, previous sentiment analysis tasks cannot fully meet the needs of users. This paper aims to study the metaphorical function and affective cognition in Internet English loanwords. This paper proposes a neural network algorithm and conducts a comprehensive analysis of the metaphorical function and emotional cognition of Internet English loanwords. The neural network algorithm has a powerful sentiment analysis function, so the article chooses this algorithm. The experimental results of this paper show that with the popularity of the Internet, more and more people go online. In 2013, the proportion of Internet users was the highest at 23.2%. In 2015, the proportion of Internet users was 38.3%, an increase of 15.1% in just one year. The percentage of people online will reach 68.3% by 2021, indicating that almost half of the people have learned to surf the Internet. This also means that Internet English loanwords have also been developed. The rapid development of loanwords in Internet English is because they have metaphorical functions and express people's emotions.

## 1. Introduction

In recent years, with the rapid development of economic globalization and information dissemination, the Internet has become more and more popular around the world as a new dissemination method. As a result, numerous Internet communication platforms, such as Sina, microblog, and Baidu Tieba, have undergone tremendous development. As a tool used by people in the network environment, the Internet catchphrase is a language used by netizens to express their own feelings and opinions. It is the carrier of information and communication in the network environment. As a special network language expression form, the network English loanwords contain a large number of metaphorical expressions. The influence of emotions on people is mainly value judgment. In layman's terms, a person's emotional cognition determines a person's values. When people have emotional resonance with something, they will have a value identification with that something.

As individuals with their own independent consciousness, human beings have their own unique emotional experience of the world. Emotional metaphor is essentially a cognitive process of metaphorizing emotion. Meanwhile, people perceive and interpret the world around them based on their own experience. The object of human perception is the perception of spatial orientation first, and then the concept of orientation is projected onto emotion and other aspects so as to obtain the concept of these things. Metaphors are an important factor in explaining the formation or structure of Internet buzzwords.

The innovation of this paper includes that: (1) This paper not only introduces the relevant theoretical knowledge of metaphor function and affective cognition but also proposes a neural network algorithm, as well as analyzes how the neural network algorithm analyzes the emotional cognition in the network of English loanwords. (2) Comparative analysis of multichannel convolutional neural networks and other algorithms are contained. Through experiments, it can be known that the multichannel convolutional neural network has a better effect on emotion classification and higher accuracy.

## 2. Related Work

With the informatization of social life and economic globalization, English has become more and more important as one of the important means of information transmission. The loanwords of Internet English have also become richer. Internet loanwords are undoubtedly not only cognitive activities but also emotional activities. Personal emotional factors will certainly affect the various stages of the Internet loanwords. People's perspectives, sentiment evaluations, and attitudes about entities and their attributes were evaluated by Niu and Huang as sentiment analysis and cognition. In sentiment analysis, vocabulary sentiment cognition has also been a hot topic. A binary relation knowledge base was created by combining the current sentiment dictionary with manual annotation for annotation. This method had the advantages of high processing speed and a low occupancy rate when compared to older methods [1]. Mammarella found that the effects of microgravity on cognition and mood have been studied separately in recent decades. He emphasized the need to focus on emotion-cognitive interactions as a framework for explaining spatial cognitive performance. He briefly analyzed the interaction between affective variables and spatial cognition. All in all, this approach showed an interesting data pattern [2]. Kensinger and Gutchess reviewed recent research on social and emotional aspects of cognitive aging and how these elements intersect in a variety of ways. He studied models for cognitive aging and how they influenced socioemotional aspects. He also found that cognitive aging models could be effectively applied to socialemotional aging [3]. Efendic et al. found that people's emotional experience could be affected by a variety of information inputs; however, it was not clear which factors were affected. He studied the construction of emotionally informative experiences and explored whether the resulting emotional experiences map to people's valuation judgments [4]. Perceived risk was discovered to be an important component of health decision theory by Klasko-Foster et al. When the emotional aspects of risk were researched as predictors of behavior, they were frequently separated from the cognitive aspects. The more intricate relationships between emotion and cognition are less studied [5]. Sern et al. discovered that people in negative affective states were more responsive to unexpected rewards than people in neutral or positive affective states, but the unexpected reward acquisition was less sensitive. When compared to exposure to rewarding stimuli, unexpected rewards elicited relatively favorable affective states in participants, suggesting that affluent surroundings are connected with positive affective states [6].

With the advent of the network information society, people have more and more opportunities to communicate through the network. The development of Internet loanwords in English is also getting faster and faster, which is loved by the majority of netizens. The Internet English loanwords are not only vocabulary but also the sustenance of the speaker's emotional expression. However, with the surge in the number of Internet users, there are more and more foreign words in Internet English. Their metaphorical function and emotional cognition are cluttered and unclear due to the huge amount of data. The metaphorical function and emotional cognition analysis of traditional Internet English loanwords can no longer meet the needs of Internet development. The above-mentioned scholars' descriptions and experiments on emotional cognition are far from enough evidence. Therefore, based on the neural network, this paper classifies the metaphorical function and emotional cognition of Internet English loanwords so as to facilitate the emotional cognition of netizens.

## 3. Metaphoric Function of Foreign Words Based on the Neural Network and Emotional Cognition

### 3.1. Development of Loanwords in the Internet English

The change of English loanwords in the Internet language to the existing language components is mainly reflected in the “form,” which uses the most concise characters to skillfully set the span of verbal communication and shorten the precious time of information communication. With the development of information technology, especially the emergence of virtual communication tools such as microblog and WeChat, the loanwords in Internet English is gradually becoming the “common language” of people who are pursuing the fashion of language communication [7]. On the Internet, in terms of loanwords, in various aspects such as technology, food, art, entertainment, life, and so on, loanwords in English are mixed in Chinese. On the other hand, young people consider that people on the Internet are the main body of Western language and cultural identity. It also reflects that people's pursuit of novelty and fashion begins with the strong vitality of English self-renewal and development [8].

Internet in China experienced explosive growth in 2013, and Internet applications have been increasingly diversified and developed in an all-round way. The prosperity of social networks has resulted in a large number of Internet buzzwords appearing every year. The percentage of people accessing the Internet in recent years is shown in Figure 1:

As shown in Figure 1, with the vigorous promotion of the Internet and its increasing use, a large number of corresponding derivative words have been born, from the original pure computer terms to today's Internet buzzwords, all of which confirm the huge impact of the Internet on the current society. In particular, the latter has the characteristics of rapid derivation and dissemination, a wide range of types, and rich content. To a certain extent, the changes in Internet buzzwords reflect the changes of a specific era, different social concerns, and emotional changes of netizens [9].

As a medium of communication platform, Internet loanwords in English promote people's communication and play an increasingly important role in people's daily lives [10]. Internet English loanwords, as a linguistic phenomenon, are more and more favored by users, especially the younger generation, due to their rich language expression and rich creativity, which inevitably has attracted the attention and interest of many researchers. The level of interest of netizens in online English loanwords is shown in Figure 2:

As shown in Figure 2, the largest percentage of people are very interested in English loanwords, and a very small percentage of people are disinterested. In Internet terms, there are about 3 types of Internet neologisms borrowed from English vocabulary. One is homophony. These words are mainly used to express personal feelings and to illustrate the objective situation in network communication. For example, “gou dai” is a transliteration of the English phrase “go die.” Another example is the transliteration of idol -- “idou.” The second is a direct translation of the word according to the meaning. For instance, the Internet term “ni zhi dao” comes from the English of “you know” and “noZUOnodie” is equivalent to the Chinese Internet catchphrase “bu zuo jiu bu hui si.” The third type is a mixed translation of Chinese and English. For example, “word tian” is equivalent to “wo de tian” in Chinese.

In fact, Internet buzzwords are not limited to words but also include phrases or sentences used in Sina, microblogs, Baidu Tieba, or forums, online chat rooms, and BBS. In addition, these phrases or expressions even include sentences frequently used by Internet users comment on certain topics or social events in cyberspace. Therefore, in this paper, the author will mainly focus on the words, phrases, and sentences that are frequently used in the abovementioned cyberspace. Internet buzzwords are widely used by Internet citizens among them.

#### 3.1.1. Metaphoric Function

As a cognitive method, conceptual metaphor theory is one of the important fields of cognitive linguistics. It plays an important role in the conceptual construction and cognition of language-developed people [11]. Initially, metaphors were considered as rhetorical devices, including similes, explicit metaphors, and loanword metaphors. Different from previous views on metaphor, conceptual metaphor theory holds that metaphor is not only a linguistic phenomenon but also a cognitive conceptual thinking process. Metaphorical thinking is very important for people to understand and experience things in daily life, and it is one of the most important ways through which a conceptual system must be established. Not only are rhetorical metaphors included in the category of cognitive metaphors, but other related rhetorical mechanisms are also included in the category of cognitive metaphors [12].

Metaphor research has always been one of the hottest topics in cognitive linguistics research. Cognitive metaphor research not only provides a cognitive method for metaphor research but also makes a leap forward in the study of rhetorical devices [13].

From a cognitive point of view, traditional metaphors, and innovative metaphors are very common in Internet buzzwords. People tend to unknowingly equate these two similar things.

*(1) Structural Metaphors*. Structural metaphors refer to the structure of one concept being used to construct another. The superposition of two concepts describes some related aspects of one concept used to talk about another concept, resulting in the phenomenon of multiple uses of a word. Structural metaphors are based on systematic connections in people's feelings and lived experiences.

*(2) Orientational Metaphors*. In the network language, there are many orientation metaphors, which are used to express people's cognition or understanding of the concept of space, such as in-out, up-down, front-back, and right-left. One could say he felt fine after being outdoors, or one could say she was upset after hearing bad news from her mother. In this expression, up and down are the source domains, and emotion is the target domain, and the relationship between the upper and lower spaces is mapped to the emotional relationship, so as to better understand human emotions. In real life, when people feel sad or depressed, they usually hang their heads and droop their eyelids. On the contrary, when people's emotions are high, their thoughts are usually high as well.

*(3) Ontological Metaphors*. Ontological metaphors are conceptual metaphors that allow people to perceive events, activities, emotions, and physical entities in relatively easy-to-understand ways. In an ontology metaphor, the concept of source domain is usually a concrete expression of physics, while the concept of target domain is a vague and abstract expression. People will have such a conceptual structure after their experience in the material world, and then they will use a set of relatively abstract fields to organize their thoughts.

There are many examples of directional metaphors and structural metaphors in Internet buzzwords. However, in the network metaphor, the third type, ontological metaphors, has the largest proportion. Class experience provides an important basis for understanding abstract conceptual representations as “entities”. In this metaphor, abstract and vague ideas, feelings, mental activities, events, states, and other intangible concepts are regarded as entities.

#### 3.1.2. Emotional Function and Emotional Factor Definition of English Loanwords in Internet Language

The relationship between emotion and memory has been corroborated by a large number of studies in related fields such as linguistics, psychology, and cognitive science. The research on emotional vocabulary, memory, and retrieval among them has made remarkable progress. Emotional words refer to words that contain emotional factors [14]. Different from happy, angry, sad, and other words that express emotions immediately, they imply emotional state in the meaning of words. With the rise and development of human psychology, the emotional issues in foreign language education have attracted more and more attention. Human psychology believes that education should be aimed at promoting people's comprehensive development. In order to achieve this goal, the two aspects of cognition and emotion must be unified.

Loanwords have an emotional function in English, which helps netizens express the most direct and richest ideological meaning in the simplest and fastest way. This not only reflects the economy, openness, and comprehensiveness of Internet terms but also meets the emotional needs of netizens.

#### 3.1.3. Emotional Cognition Based on Deep Learning

Deep learning involves learning the underlying principles and levels of representation of sample data, and the knowledge acquired during these learning processes is very useful for interpreting data types like text, images, and sounds. Deep learning's ultimate goal is to give machines the capacity to analyse, learn, and recognise information like text, images, and sounds. In a deeper emotional cognitive analysis task compared with the usual emotional analysis, it is necessary to consider the emotional information of various targets or aspects in the text when entity targets and specific aspects for emotional analysis are used. Because short texts usually do not follow grammatical rules, have short lengths, and contain very limited information, it is difficult to directly apply traditional emotion classification models to the emotional cognitive analysis task of short texts.

With the development of deep learning technology, emotion analysis models based on deep networks have recently achieved outstanding success. Deep learning [15, 16] has made significant advances in a variety of fields, including image processing [17], audio recognition, robotics, natural language processing [18, 19], and others. Deep learning-based sentiment classification models have outperformed more conventional techniques in sentiment analysis, and they do so without overly relying on feature engineering.

### 3.2. Application of Convolutional Neural Networks in Emotional Cognitive Tasks

A feedforward neural network with a deep structure that uses convolutional computation is referred to as a “convolutional neural network” (CNN) [20]. It represents deep learning in one of its representative algorithms. Additionally, it has representation learning capabilities. Convolutional neural networks (CNNs) have received a lot of attention because they are widely used in many fields and because they do not require a significant amount of preprocessing work in the task. This effectively reduces the need for feature engineering.  Figure 3 depicts the model's structure for the convolutional neural network.

The input layer, convolutional layer, pooling layer, and fully connected layer are the four layers that make up the majority of the CNN, as shown in Figure 3. The most crucial information expression in tasks involving natural language processing is found in the word features of text. Through an input layer, the CNN receives text word vector representations [20]. The network model's input layer matrix is represented by the following formula for a sentence of length *n*:

(1) $$\begin{array}{c} a_{1:n}\in R^{n\times k}. \end{array}$$

Obtaining the convolutional feature vector of the input information in the following formula:

(2) $$\begin{array}{c} c=f\left(W\cdot a+b\right). \end{array}$$

In formula (2), *W* is the weight matrix; *b* is the bias; *f* is the activation function.

A deep feedforward neural network with weight sharing and local connections is the convolutional neural network (CNN). The convolutional neural network CNN was first primarily used to process image data, but later researchers used it to perform text classification. In the sentiment analysis task, sentiment feature information directly affects the sentiment polarity judgment of the text. Convolutional neural networks can also combine word vectors and sentiment features into network inputs to construct classification patterns [21]. The CNN sentiment analysis model is shown in Figure 4:

As shown in Figure 4, CNN performs feature extraction learning on the input sentence by receiving the word vector and sentiment feature vector of the text. For a sentence of length *n*, the input vector is represented by the following formulas:

(3) $$\begin{array}{c} e_{1:n}=e_{1}⊕e_{2}⊕\cdots ⊕e_{n}, \end{array}$$

(4) $$\begin{array}{c} e_{i}=a_{i}⊕{\text{sent}}_{i}. \end{array}$$

In formulas (3) and (4), *a*_*i*_ is the word vector and sent_*i*_ is the sentiment feature. As shown in the following formula:

(5) $$\begin{array}{c} C=\left[c_{1},c_{2},\ldots ,c_{n-l+1}\right]. \end{array}$$

The *c*_*i*_ extracted from the component *e*_*i*:*i*+*l*−1_ after the convolution operation is as shown in the following formula:

(6) $$\begin{array}{c} c_{i}=f\left(w\cdot e_{i:i+l-1}+b\right). \end{array}$$

The convolution kernel weight is represented by *w* ∈ *R*^*l*×(*m*+*k*)^. The pooling operation can be used to extract the most important feature information of the input sentence as shown in the following formula:

(7) $$\begin{array}{c} \overset{\wedge }{c}=\max\left\{C\right\}. \end{array}$$

The result obtained by convolution kernel sampling is $\overset{\wedge }{c}$, and the feature information sampled by *k* convolution kernels can be expressed as shown in the following formula:

(8) $$\begin{array}{c} C=\left[{\overset{\wedge }{c}}_{1},{\overset{\wedge }{c}}_{2},\ldots ,{\overset{\wedge }{c}}_{k}\right]. \end{array}$$

The fully connected layer receives the feature information sampled by the pooling layer as an input, and the classification result is obtained as shown in the following formula:

(9) $$\begin{array}{c} b=\text{soft}\max\left(W_{f}\cdot C+B_{f}\right). \end{array}$$

In formula (9), *W*_*f*_ ∈ *R*^*d*^ is the weight of the fully connected layer; *B*_*f*_ ∈ *R* is the bias; *b* is the output result.

### 3.3. Application of Long- and Short-Term Memory (LSTM) Network in Sentiment Task

A type of time-recurrent neural network called the long- and short-term memory network was created specifically to address the general RNN's long-term dependence issue (recurrent neural network). A superior version of the neural networks used today is the long- and short-term memory (LSTM) network (RNN). It may successfully address the issue of gradient vanishing in conventional network training while maintaining the long-term dependability of the input data according to Figure 5:

Figure 5 illustrates how the more widely used LSTM—long- and short-term memory network—is an improved recurrent neural network that can address the issue that RNN cannot handle long-distance dependencies. Memory cells are used by the LSTM network to store and save key input sentence feature data. Additionally, there are instances where irrelevant information is overlooked. A core unit and three unique gate units make up each neuron. The LSTM unit determines the new contextual memory information as shown in the following formula by combining the input from this time with the output from the hidden layer from the previous time:

(10) $$\begin{array}{c} {\tilde{c}}_{t}=\tanh\left(W_{c}a_{t}+U_{c}h_{t-1}\right). \end{array}$$

The output of the hidden layer at time *h*_*t*−1_ is shown in the following formula:

(11) $$\begin{array}{c} c_{t}=f_{t}c_{t-1}+i_{t}{\tilde{c}}_{t}. \end{array}$$

In natural language processing tasks, the LSTM receives the input of text serialization, fully considering the temporal relationship between words. It also mines the dependencies between words in the input text and learns the long-term dependencies of words in the text. The LSTM sentiment analysis model is shown in Figure 6:

As depicted in Figure 6 the word vector is used as the network input in the LSTM sentiment analysis model. Each LSTM unit's input comprises of the output of the previous unit's hidden layer, as well as the word vector input this time. At time *t*, the hidden layer's output as shown in the following formula :

(12) $$\begin{array}{c} x_{h}^{t}=\sum_{i}^{E}w_{ih}e_{i}^{t}+\sum_{h^{\prime }}^{H}w_{h^{\prime }h}y_{h^{\prime }}^{t-1}. \end{array}$$

In formula (12), *e*_*i*_^*t*^ is the word vector. Finally, a softmax function is used to receive the last hidden layer output of LSTM. Then the classification result is obtained as the following formula :

(13) $$\begin{array}{c} b=\text{soft}\max\left(Wy^{T}+B\right). \end{array}$$

In formula (13), *y*^*T*^ is the output of the hidden layer at the last time step; *W* is the weight matrix; *B* is the bias.

### 3.4. Emotional Cognitive Model Based on Multichannel CNN

By using convolution kernels of various sizes, the sentiment classification model based on convolutional neural networks (CNN) extracts rich features from the input text and can fully mine the emotional feature information in the text. Without extensive feature engineering, it can produce better sentiment classification results than conventional machine learning techniques. Some studies combine word vectors with emotional feature data specific to sentiment analysis tasks as the input of CNN in the short-text sentiment analysis task because of the limited information contained in the short-text. This allows them to extract richer emotional features from texts so that deeper hidden emotional feature information in short texts can be mined.

This chapter introduces the MCCNN, a multichannel convolutional neural network model that takes into account both word position features and emotional part-of-speech characteristics. In order to efficiently obtain the emotional feature information of the input sentence during the training process, the model builds a text input matrix for the specific emotional information needed for the sentiment analysis task.  Figure 7 shows the multichannel convolutional neural network model's structure:

As shown in Figure 7 MCNN model forms various network input channels through the combination and transformation of various functions. Therefore, the model can obtain richer emotional functional information based on various information from various input channels. The combination of different feature vectors can not only form new features but also allow the model to learn the relationship and influence between features. The MCNN model enables the network model to complete the adjustment and optimization of various feature vectors in one learning process by simultaneously receiving input information from various channels.

#### 3.4.1. Sentiment Feature Construction of Foreign Words

Convolutional neural networks need to receive parallel inputs of text at a time. For each sentiment score, this chapter represents the score value as a multidimensional continuous value vector, as shown in the following formula :

(14) $$\begin{array}{c} es_{i}=\left[e_{1},e_{2},\ldots ,e_{p}\right]. \end{array}$$

Here *p* is the vector dimension. In the same way, for the weighted score for each common term, as shown in formula (15), the weighted score is mapped into a multidimensional continuous-valued vector of the same dimension.

(15) $$\begin{array}{c} ew_{i}=\left[e_{1},e_{2},\ldots ,e_{p}\right]. \end{array}$$

Here *ew* ∈ *R*^*p*^ is a vector representation.

#### 3.4.2. Model Training

This chapter uses different convolutional layers to extract the feature information of the input text. For a convolution kernel of length *l*, the convolution operation is as in the following formula:

(16) $$\begin{array}{c} c_{j}=\text{relu}\left(W\cdot V_{j}^{i:i+l-1}+b\right), \end{array}$$

ReLu is the activation function used in the experiments in this chapter. The feature map can be obtained through the convolution operation, as shown in the following formula:

(17) $$\begin{array}{c} c=\left[c_{1},c_{2},\ldots ,c_{n-l+1}\right]. \end{array}$$

The pooling layer takes the maximum value of each feature map in a max-over-time pooling method to obtain a 300-dimensional vector. Max-over-pooling can solve the variable-length sentence input problem. For the feature vector map of each channel, the pooling layer adopts the max-over-time pooling method to downsample. As shown in the following formula :

(18) $$\begin{array}{c} \overset{\wedge }{c}=\max\left[c\right]. \end{array}$$

In the multilevel feedforward neural network, the hidden layer refers to the layers other than the input layer and the output layer. It is not possible for the hidden layer to directly send or receive signals from the outside world. It is only required when the data are separated nonlinearly. This chapter uses a hidden layer to learn and adjust the feature vectors obtained from different input channels, as shown in the following formula:

(19) $$\begin{array}{c} R=\text{relu}\left(W_{h}\overset{\wedge }{C}+y_{h}\right). \end{array}$$

In the following formula , *W*_*h*_ is the weight matrix, *y*_*h*_ is the bias. The optimized network model is shown in the following formula:

(20) $$\begin{array}{c} \text{loss}=-\sum_{i\in D}\sum_{j\in C}b_{i}^{j}+\lambda {\left\|\theta \right\|}^{2}, \end{array}$$

*b*_*i*_^*j*^ is the actual category. *λ*‖*θ*‖^2^ is the regular term.

## 4. Experiment of Emotion Cognition Based on Multichannel Convolutional Neural Network

### 4.1. Experiment on the Accuracy of Sentiment Classification Based on Multichannel Convolutional Neural Network

From the COAE2014 dataset, 200 pieces of data with emotional polarity are extracted as training and test sets, including 98 positive emotional words and 102 negative emotional words. Furthermore, in order to verify the strong robustness of the MCNN model, a hybrid dataset was made by extracting 100 emotional data from the dataset. Detailed data statistics are shown in Table 1.

As shown in Table 1 this paper compares the proposed model method with the widely used traditional machine learning method and the deep network model method. The article also analyzes the classification accuracy, training time, and model robustness of each model in the sentiment analysis task. The comparison models are SVM and traditional SVM and CNN. Among them, the SVM classifier is combined with the emotion analysis task through a relational target to achieve better emotion classification results than previous machine learning methods.

Because better sentiment classification results can be achieved through multichannel input methods, the SVM, CNN, and LSTM models proposed in this chapter and the MCCNN are used for two-class comparison experiments. The classification accuracy rates of the four models on different data sets are counted as shown in Table 2:

As shown in Table 2 the MCNN model proposed in this chapter achieves the highest sentiment classification results in all three datasets. Compared with 80.53% of the CNN model and 83.08% of the SVM model, the classification positive solution rate of the highest MBD dataset is 85.70%, with an increase of 5.7% and 2.62%, respectively.

In order to further verify that the MCCNN model proposed in this chapter can mine more hidden features, 150 samples were randomly selected from the COAE and MBD datasets to conduct 10-fold cross-validation experiments on the MCCNN model proposed in this chapter and the comparison method. The comparison results are shown in Table 3.

As shown in Table 3, the MCCNN model achieved the best emotion recognition classification effect on both datasets, with classification accuracy rates of 92.31% and 93.35%, respectively, showing that it can achieve a better emotional classification effect, which verifies the robustness of the MCCNN model. It indicates that the MCCNN model that uses multiple channels to receive text feature input can mine more hidden feature information from different forms of feature representations. Therefore, the effect of sentiment classification is more advantageous than other models.

### 4.2. Experiments on Sentiment Based on Multichannel Convolutional Neural Network in Different Dimensions

This paper compares the SVM, CNN, LSTM, and MCCNN models using different dimensions of part-of-speech features to analyse whether it will affect the sentiment classification effect of the model. The experimental results are shown in Figure 8:

As shown in Figure 8 when the dimension of part-of-speech features is greater than 30, the classification effect of the CNN and LSTM models decreases with the increase in dimension. The MCNN model with location features has better classification performance than the CNN and LSTM models, which shows that location features can improve the classification accuracy of the model.

In order to compare whether SVM, CNN, LSTM, and MCNN models use word vectors of different dimensions to affect the effect of sentiment classification, this paper conducts experimental analysis as shown in Figure 9:

As shown in Figure 9 when the word vector dimension value exceeds 30, the classification accuracy of SVM, CNN, and LSTM starts to stop rising, while the MCNN model will continue to rise.

## 5. Conclusion

With the gradual improvement of China's Internet utilization, people's communication methods have changed from the previous single type to novel and diverse types, all showing the strong power of the Internet itself. The characteristics of the Internet's all-weather, wide dissemination, and many participating groups have solved the information asymmetry to the greatest extent. The power of Internet includes the power of technology, communication, Internet companies, and netizens. If this power becomes a combined force, it will be a huge energy to overcome difficulties. Meanwhile, people's communication languages are more abundant. The network language adds color to people's daily communication due to its entertainment, rapidity, novelty, and other characteristics. Among them, Internet English loanwords have become a popular Internet catchphrase. It not only has the function of metaphor but also can represent people's emotional expression. However, in the previous analysis of the metaphorical function and emotional cognition of loanwords in Internet English, the emotion of loanwords cannot be effectively classified. Therefore, this paper proposes a method of emotion recognition classification based on neural networks. In the method part, a brief exposition is made on why neural networks are chosen to classify emotion cognition. In the experimental part, this paper conducts experiments and analysis on the sentiment classification function of the multichannel convolutional neural network and compares it with various classification methods. Finally, it is found that the sentiment classification efficiency of the multichannel convolutional neural network is higher and its accuracy is also higher.

## Figures and Tables

**Figure 1:** Percentage of Internet access in recent years.

**Figure 2:** Netizens' interest in online English loanwords.

**Figure 3:** Convolutional neural network model structure diagram.

**Figure 4:** CNN sentiment analysis model.

**Figure 5:** LSTM network unit structure.

**Figure 6:** LSTM sentiment analysis model.

**Figure 7:** Multichannel convolutional neural network model structure.

**Figure 8:** Comparison of part-of-speech features in different dimensions.

**Figure 9:** Comparison of word vectors of different dimensions.

**Table 1:** Experimental data statistics.

Data set	Corpus	Positive sample size	Negative sample size
COAE-train	COAE2014	25	27
COAE-test	COAE2014	25	27
MBD-train	MBD	17	15
MBD-test	MBD	18	10
COAEMBD-train	COAE2014 + MBD	9	16
COAEMBD-test	COAE2014 + MBD	5	7

**Table 2:** Comparison of sentiment classification performance of different models.

Model	Correct rate		
	COAE	MBD	COAEMBD
SVM	0.8125	0.8308	0.8041
CNN	0.7644	0.8053	0.7520
LSTM	0.8295	0.8262	0.7993
MCCNN	0.8476	0.8570	0.8421

**Table 3:** Cross-validation experimental results.

Model	Correct rate	
	COAE	MBD
SVM	0.8901	0.8937
CNN	0.8962	0.8995
LSTM	0.9037	0.9076
MCCNN0.923	0.9231	0.9335

## Data Availability

The data used to support the findings of this study are available from the corresponding author upon request.
